# Treatment of intra-bony defect and periodontal phenotype modification therapy (PhMT): A one-year follow-up case report

**DOI:** 10.1097/MD.0000000000041191

**Published:** 2025-01-03

**Authors:** Ali Fahed Alqahtani

**Affiliations:** a Department of Periodontics and Community Dentistry, College of Dentistry, King Khalid University, Abha, Kingdom of Saudi Arabia.

**Keywords:** allografts, case report, guided tissue regeneration, intra-bony defect, periodontitis

## Abstract

**Rationale:**

The treatment of a patient with an intrabony defect using periodontal phenotype modification therapy (PhMT) is alternative approach in correcting intrabony defects and changing periodontal phenotypes.

**Patient concerns:**

A 27-year-old male patient arrived with a severe intrabony defect and a poor periodontal phenotype. The patient received PhMT, which includes nonsurgical periodontal therapy, bone grafting, and orthodontic treatment. After 1 year, there were considerable changes in the intrabony defect, periodontal phenotype, and general oral health.

**Diagnoses:**

A 27-year-old male patient had a profound intrabony defect (10 mm) and a poor periodontal phenotype (thin gingiva, high frenum attachment).

**Interventions:**

The patient received PhMT, which includes nonsurgical periodontal therapy (scaling and root planing), bone grafting (allograft), and orthodontic treatment (correcting tooth placement). After 1 year, there were considerable improvements: Intrabony defect reduction (from 10 to 3 mm), improved periodontal phenotype (thickened gingiva, decreased frenum attachment), and improved dental health (lower pocket depths, increased attachment levels). PhMT successfully repaired the intrabony deficiency and altered the patient’s periodontal phenotype.

**Outcomes:**

Improved dental health and aesthetics were the result of the comprehensive treatment, which addressed the problem as well as the patient’s underlying periodontal features.

**Lessons:**

The efficacy of PhMT in correcting intrabony abnormalities and altering periodontal phenotypes is demonstrated in this case study. This strategy presents a viable remedy for patients with intricate periodontal requirements.

**Key points**

- Bone grafting and regenerative therapies, have shown variable success rates and often require multiple surgical interventions.
- Advances in periodontal therapy have highlighted the importance of considering the patient’s periodontal phenotype in treatment planning.
- Periodontal phenotype modification therapy is a comprehensive approach that aims to modify the patient’s periodontal characteristics, such as gingival thickness and frenum attachment, to improve treatment outcomes.

## 1. Introduction

### 1.1. Background

Untreated periodontal disease can result in tooth loss because it is a chronic inflammatory illness. Treatment of intra-bony abnormalities is essential for achieving periodontal stability as they are a common result of periodontal disease. Reduction of pocket depth and regrowth of bone are common goals of conventional periodontal therapy. Nonetheless, the patient’s periodontal phenotype may have an impact on the result.^[1]^

A typical side effect of periodontal disease is the loss of alveolar bone and attachment apparatus due to periodontal intra-bony abnormalities. These flaws can result in tooth loss and impaired oral function, which makes them a major obstacle to periodontal care. Conventional therapeutic modalities, like bone grafting and regenerative therapies, frequently call for several surgical procedures and have varying success rates.^[2]^

### 1.2. Rationale and knowledge gap

An exceptional chance to assess the efficacy of periodontal phenotype modification therapy (PhMT) in treating a patient with a deep intra-bony defect and an unfavorable periodontal phenotype is provided by this case report. As part of PhMT, the patient received multidisciplinary care that included bone grafting, orthodontic treatment, and nonsurgical periodontal therapy. This case report’s objectives are to record the treatment results and assess how well PhMT works to achieve periodontal regeneration and phenotypic alteration throughout the course of a 1-year follow-up period.^[3]^

Our goal in publishing this case report is to add to the increasing amount of information that shows PhMT can be a successful treatment for patients with complicated periodontal requirements. Our findings will guide future research approaches in periodontal regeneration and phenotypic alteration and offer insights into the possible advantages and disadvantages of PhMT.^[1,2]^

The relevance of taking the patient’s periodontal phenotype into account while planning treatment has been brought to light by recent advancements in periodontal therapy. PhMT is a comprehensive strategy designed to improve treatment outcomes by modifying the patient’s periodontal features, such as frenum attachment and gingival thickness. PhMT modifies the periodontal phenotype through orthodontic and periodontal therapies, improving treatment results.^[2,3]^

Although PhMT has showed promise, nothing is known about how well it works in the long run to correct intra-bony abnormalities. This case report presents a 1-year follow-up of a patient treated with PhMT for an intra-bony defect in an effort to close this knowledge gap.^[3]^

Pasqualini E et al (2024) performed a systematic review to examine clinical periodontal measurements posttreatment with minimally invasive surgical technique (MIST), modified-MIST, and/or various papilla preservation techniques like entire papilla preservation, modified-papilla preservation technique, or simplified-papilla preservation technique. The results of the research showed that procedures like MIST, modified-MIST, and papilla preservation can successfully treat periodontal disease in regions with intra-bony defects with low levels of morbidity.^[4]^

A novel root coverage (RC) technique called the mixed-thickness tunnel access technique was presented by Marques T et al in their case series in 2023. It aims to augment soft tissues coronal to the gingival boundary and approaches a full-split design. According to the case series’ findings, the mixed-thickness tunnel access technique is a simpler method for minimally invasive surgical procedures, making it a viable choice for treating RC with a high success rate, predictability, and preservation of aesthetics. As a result, using the full-split design process has a technical sensitivity.^[5]^

### 1.3. Objective

This case report’s goals are to outline the PhMT therapy of an intra-bony defect and assess how well it worked over a 1-year period to achieve periodontal stability and phenotypic alteration. The purpose of this paper is to advance knowledge about PhMT’s potential for treating periodontal disease and provide guidance for future research efforts.^[1]^

## 2. Case presentation

### 2.1. Patient information

A 27 years old female patient with no relevant medical history visited the Department of Periodontics and Community Dentistry in the month of August 2023, presented with thin gingival phenotype and root prominence at lower anterior teeth. No past relevant interventions reported by the patient. The patient’s overall appearance, vital signs were normal. Findings from the head, neck, chest, lungs, and abdomen, heart sounds, and pulse were also.

### 2.2. Clinical examination

The clinical examination reveals a case of generalized chronic periodontitis characterized by deep periodontal pocket 7 mm distal to #41 with bleeding on probing and grade 1 mobility, recession type-2 recession was detected at #41, 42. A notable intra-bony defect, measuring 10 mm, is observed in the mandibular anteriors, indicating advanced periodontal destruction. The patient’s periodontal phenotype is marked by thin gingiva, high frenum attachment, and inadequate keratinized tissue, which may contribute to the complexity of periodontal management and the overall stability of the periodontal tissues.

### 2.3. Radiographic examination

The radiographic examination, including periapical radiographic examination, intra-bony defect distal to #41 was detected demonstrating significant bone loss around the mandibular anterior region, highlighting the extent of periodontal destruction in this area. Further evaluation with a cone beam computed tomography (CBCT) scan provided a detailed assessment, confirming the presence of a deep intra-bony defect. The CBCT imaging offered a comprehensive view of the defect’s depth and extent, aiding in the accurate diagnosis and planning of appropriate periodontal treatment strategies.

### 2.4. Diagnosis

By summarizing the thorough gingival and periodontal examination clinical findings, the case was diagnosed as periodontitis stage 3 grade B.

### 2.5. Treatment

#### 2.5.1. Treatment plan

Ethical approval was waived, as it is the case report and good clinical practice guidelines followed and the patient informed consent was taken before the treatment procedure. In order to properly address the patient’s periodontal problems, the suggested treatment plan includes a number of essential elements. Scaling and root planning are examples of nonsurgical periodontal therapy procedures used to eliminate plaque and tartar from tooth surfaces and lessen inflammation caused by the disease. In order to promote healing and improve bone regeneration, bone grafting using an allograft material was carried out to correct the profound intra-bony defect. Furthermore, it was advised to have orthodontic treatment to realign teeth, which can improve the stability and general health of the periodontal tissues. PhMT was used to enhance the gingival thickness and augment keratinized tissue in order to further improve the periodontal phenotype. This reduced vulnerability to future periodontal breakdown and supported long-term periodontal health.

#### 2.5.2. Treatment procedure

To ensure patient comfort and successfully address the deposition of calculus and plaque, nonsurgical periodontal therapy was performed under local anesthesia as the first step in the treatment procedures. Six weeks after the healing period, bone grafting with guided tissue regeneration was performed to assist the periodontal tissue restoration and restore the intra-bony defect. In this case study, orthodontic therapy was started 3 months before bone grafting in order to improve the periodontal environment and straighten the teeth. In addition, during the course of the treatment, PhMT was carried out to promote gingival thickness and increase keratinized tissue, which in turn improved overall periodontal health and stability Figure 1.

**Figure 1.** Showing the steps of surgical procedure: (A) Preoperative image; (B) Incision; (C) Flap elevation; (D) Degranulation; (E) Intra-bony defect depth; (F) Subepithelial connective tissue graft harvested; (G) Trap door approximation; (H) Suturing donor site; (I) Allograft mixed with I-PRF; (J) Sticky bone; (K) Graft placement at the defect; (L) Stabilization with membrane; (M) Placement of subepithelial connective tissue graft; (N) Stabilized by suture; (O) Suturing done; (P) 1 week follow-up; (Q) 2 week follow-up; (R) 1 year follow-up; (S) 1 year follow-up lingual view.

#### 2.5.3. Follow-up

In order to track progress and make sure the interventions were working, the patient was scheduled for follow-up appointments 3, 6, and 12 months after starting therapy. Clinical and radiographic assessments were performed at every follow-up appointment to evaluate the stability of orthodontic corrections overall, the success of bone graft integration, and improvements in periodontal health. These assessments yielded vital information on the healing process, enabling prompt modifications to the treatment regimen and guaranteeing the best possible long-term results.

#### 2.5.4. Clinical outcome

There was a noticeable improvement in the clinical outcomes at the 12-month follow-up. The more advantageous 2 to 3 mm range of probing depths was observed after the initial 6 to 10 mm range, suggesting that periodontal pockets had been effectively resolved. Significant improvement in attachment levels was seen, resulting in an increase of 4 to 6 mm, which is indicative of improved periodontal support. The gingival thickness increased significantly from 0.5 to 2.5 mm, which strengthened the periodontal environment. Furthermore, the gingival tissues’ stability and vitality are further supported by the growth in keratinized tissue from 1 to 4 mm. These results highlight how well the all-encompassing treatment approach worked to improve overall tissue quality and restore periodontal health.

#### 2.5.5. Radiographic outcomes

Based on a CBCT scan, the radiographic results at 12 months showed notable improvements. Effective bone regeneration and repair was demonstrated by the successful reduction of the deep intra-bony defect, which measured 10 mm originally, to 3 mm. Furthermore, there was a significant 25% increase in bone density in the afflicted area as compared to baseline values. The success of the bone grafting process and the general improvement in bone structure and density are reflected in these radiography results, which support the stability and long-term prognosis of the periodontal therapy Figure 2.

**Figure 2.** (A) Pre-periapical radiograph showing the bone reduction in the mandibular anterior region (20%–30%); (B) Pre-3D scan CBCT; (C) Post-periapical radiograph showing bone fill; (D) Postoperative 3D scan CBCT. CBCT = cone beam computed tomography.

#### 2.5.6. Periodontal phenotype modification

By the 12-month mark, the periodontal phenotypic modification had produced noticeable improvements. The gingival thickness grew from 0.5 to 2.5 mm, a 400% increase that markedly improved tissue support and resilience. Additionally, there was a noticeable 300% increase in keratinized tissue, from 1 to 4 mm, which helped to create a gingival environment that was more stable and protective. Furthermore, a 2 mm reduction in the high frenum attachment was accomplished, which lessened its influence on the periodontal tissues and enhanced the overall periodontal phenotype. Together, these changes strengthened the gingival structure and improved periodontal health.

#### 2.5.7. Orthodontic outcomes

Significant improvements were observed in the orthodontic outcomes during the 12-month follow-up. Significant progress was made in tooth location, leading to better alignment and spacing and a more aesthetically acceptable and practical dental arrangement. Significant progress was also shown in the bite connection, where a more ideal occlusal relationship was formed, improving comfort and function. In addition to complementing the overall periodontal therapy, these beneficial improvements in orthodontic alignment and occlusion also help to create a more balanced and healthy dental environment.

#### 2.5.8. Patient-reported outcomes

Patient-reported outcomes at the 12-month point show a significant improvement in oral health-related quality of life, with a 50% improvement reported. This notable improvement shows how the patient’s everyday functioning and general well-being have improved as a result of the thorough treatment. The patient also showed a great deal of satisfaction with the results of the treatment, demonstrating how well the therapeutic approaches addressed both functional and aesthetic concerns. These outcomes highlight how well the treatment plan worked to improve the patient’s quality of life and happiness with their dental health in addition to meeting clinical and radiographic goals Figure 3.

**Figure 3.** Showing the timeline of sequence of treatment procedures performed.

## 3. Discussion

### 3.1. Key findings

In addressing a deep intra-bony lesion and changing the periodontal phenotype, the current case study highlights the efficacy of PhMT. Clinical, radiographic, and patient-reported results were significantly improved as a result of the treatment plan, which included nonsurgical periodontal therapy, bone grafting, orthodontic treatment, and PhMT.^[6]^

The increase in attachment levels and decrease in probing depths are in line with earlier research on regenerative periodontal therapy. But the notable improvements in frenum attachment and gingival thickness and keratinized tissue demonstrate how well PhMT works to alter the periodontal phenotype.^[7]^

This case report presents a novel application of orthodontic treatment to improve periodontal phenotype and correct tooth location. Most likely, the enhanced occlusal connection and tooth alignment played a role in the overall effectiveness of the therapy.^[6,7]^

The significance of taking patient-centered outcomes into account in periodontal therapy is shown by the patient-reported outcomes, which include enhanced oral health-related quality of life and high satisfaction. This case report’s short follow-up period and single-case methodology are 2 of its limitations. Larger sample numbers and longer follow-up times should be the goals of future research in order to confirm PhMT’s efficacy.

### 3.2. Comparison with similar researches

In 2020, Cortellini P et al carried out a study comparing the professional, patient-reported, and economic effects of periodontal regeneration against tooth extraction and replacement in a population with attachment loss to or beyond the apex of the root. According to the study’s findings, periodontal regeneration is a less expensive option than having teeth extracted and replaced, and it can improve the prognosis of teeth that are in terminal condition. Although the treatment’s intricacy prevents it from being widely used to the most complicated patients, it offers compelling evidence of the benefits of periodontal regeneration in profound intra-bony defects.^[7]^

In order to bring those consensus reports up to date, Kao RT et al^[8]^ carried out a systematic review in 2015, examining surgical techniques, biologics, and patient-, tooth-, and site-centered factors in the context of periodontal regeneration approaches developed for the correction of intra-bony defects. The review’s findings showed that biologics—a derivative of the enamel matrix and recombinant human platelet-derived growth factor-BB plus β-tricalcium phosphate—are generally better than open flap debridement procedures in terms of improving clinical parameters when treating intra-bony defects, and they are comparable to demineralized freeze-dried bone allograft and GTR.^[9]^

In 2019, Rahman A et al^[10]^ carried out a study to compare control teeth to the stability of attachment attained in infra-bony defects by regeneration treatment over 60 ± 12 months. According to the study’s findings, PAL-V obtained through regenerative therapy in cases with infra-bony deficiencies is just as stable over a 5-year period as gingivitis or periodontally decreased but healthy gingiva. The recurrence of periodontitis and smoking are linked to attachment loss.^[11]^

In order to determine whether PhMT, which involves either soft tissue augmentation (PhMT-s) or hard tissue augmentation (PhMT-b), offers therapeutic benefits for patients receiving orthodontic treatment, Wang CW et al^[12]^ conducted a comprehensive study in 2020. According to the study’s findings, PhMT-b, when combined with corticotomy-assisted orthodontic therapy through particulate bone grafting, may have therapeutic advantages in the form of altered periodontal phenotype, preserved or increased facial bone thickness, accelerated tooth movement, and increased range of safe tooth movement for patients undergoing orthodontic tooth movement.^[13]^

Based on clinical and radiographic criteria, Haripriya N et al^[3]^ study from 2024 compared and assessed the efficacy of demineralized freeze-dried bone allograft (DFDBA) versus titanium-prepared platelet-rich fibrin (T-PRF) in treating intra-bony defects. In intragroup comparisons, there were statistically significant differences in baseline values to 9 months for both “T-PRF and DFDBA groups” clinical and radiographic data. According to the study’s findings, T-PRF has demonstrated effective outcomes for treating intra-bony periodontal abnormalities that are on par with DFDBA.^[14]^

Despite having a poor prognosis, Kahn S et al^[4]^ case report from 2022 showed how a difficult clinical case was handled using a multidisciplinary strategy to ensure its maintenance. It was linked to endodontic therapy using mucogingival methods, like dental connective tissue grafting and periodontal microsurgery. The clinical significance of this case report is that, particularly in difficult cases, the outcome may be directly impacted by the appropriate diagnosis and technique choice. Despite the bad prognosis, a high degree of RC, aesthetic recovery, and a satisfactory conclusion may be achieved with the support of a good treatment plan, patient participation, and technique expertise.^[15]^

To evaluate the effectiveness of macro- and microsurgical techniques in removing the epithelial tissue layer of subepithelial connective grafts extracted using the parallel incision method, Kahn S et al carried out a pilot randomized controlled experiment in 2021.^[5]^ According to the study’s findings, samples taken by microsurgery showed identical connective layer thickness and larger residual epithelium sections than samples taken by macrosurgery.^[16]^

In 2022, Simões-Pedro M et al,^[6]^ compared the mechanical characteristics using tensile strength and examined the structural arrangement of membranes made using the original protocols of L-PRF (leukocyte platelet-rich fibrin), A-PRF (advanced platelet-rich fibrin), and A-PRF+ which differed in centrifugation speed and duration. According to the study’s findings, A-PRF + generated membranes with notable and elevated maximum traction results, suggesting superior viscoelastic strength when subjected to 2 opposing pressures.^[17]^

### 3.3. Implications and actions needed

When correcting deep intra-bony abnormalities, PhMT can be a useful supplement to conventional regenerative periodontal therapy.^[10,12,17,18]^

PhMT can enhance periodontal phenotype, which will enhance patient satisfaction and treatment results.

In order to improve periodontal phenotype and tooth location, orthodontic treatment can be a beneficial adjunct to complete periodontal therapy.^[19,20]^

## 4. Conclusions

This case study illustrates how PhMT can effectively cure a deep intra-bony lesion and change the periodontal phenotype. The all-encompassing treatment strategy, which included PhMT, bone grafting, orthodontic therapy, and nonsurgical periodontal therapy, produced notable improvements in clinical, radiological, and patient-reported results. This case report demonstrates the potential of PhMT to enhance treatment outcomes in periodontal regeneration and phenotypic alteration, despite certain restrictions. To confirm these results and make PhMT the accepted standard of care in periodontal therapy, more investigation is required. Clinicians can enhance patient outcomes and quality of life by using an all-encompassing, multidisciplinary strategy.

## Author contributions

**Conceptualization:** Ali Fahed Alqahtani.

**Data curation:** Ali Fahed Alqahtani.

**Formal analysis:** Ali Fahed Alqahtani.

**Investigation:** Ali Fahed Alqahtani.

**Methodology:** Ali Fahed Alqahtani.

**Project administration:** Ali Fahed Alqahtani.

**Supervision:** Ali Fahed Alqahtani.

**Validation:** Ali Fahed Alqahtani.

**Writing—original draft:** Ali Fahed Alqahtani.

**Writing—review & editing:** Ali Fahed Alqahtani.
